RETRACTED

# Comprehensive Rehabilitation Therapy Plus Glucosamine Hydrochloride for Exercise-Induced Knee Injuries and the Effect on Knee Function of Patients

**DOI:** 10.1155/2022/8120458

**Published:** 2022-06-27

**Authors:** Na Liu, Binggang Wang

**Affiliations:** Orthopaedics Department, The Second Hospital of Tangshan, Tangshan, China

## Abstract

**Objective:**

To assess the application value of comprehensive rehabilitation therapy plus glucosamine hydrochloride for exercise-induced knee injuries and its effect on knee function.

**Methods:**

A total of 96 patients with an exercise-induced knee injury who were admitted to our hospital from February 2019 to February 202 were recruited and assigned at a ratio of 1 : 1 with matched general information to a control group (*n* = 45) or an experimental group (*n* = 51). Both groups of patients received comprehensive rehabilitation therapy, and the patients in the experimental group were daily given additional glucosamine hydrochloride tablets for 8 weeks.

**Results:**

The experimental group showed a higher treatment efficacy than the control group (*P* < 0.001). After the treatment, the VAS scores and C-reactive protein of the two groups showed a decline, with a lower result in the experimental group than in the control group (*P* < 0.001). The Lysholm knee scores were increased in the two groups after the treatment, and the experimental group had a higher score (*P* < 0.001). After the treatment, patients of both groups showed reduced five-times-sit-to-stand-test (FTSST) results, with a better outcome obtained in the experimental group (*P* < 0.001).

**Conclusion:**

Comprehensive rehabilitation therapy plus glucosamine hydrochloride effectively improves the clinical efficacy of exercise-induced knee joint injuries and enhances the knee joint rehabilitation of the patients.

## 1. Introduction

The ligament structure of the knee joint, in the middle of the lower limbs and between the two largest lever arms of the body, is crucial in maintaining the stability of the knee joint. Knee injuries are extremely common during sports, mainly manifesting as ligament and meniscus injuries [1–4], and related symptoms include joint pain, swelling, effusion, locked knee, and quadriceps atrophy. Currently, comprehensive rehabilitation therapies such as massage, acupuncture, and traditional Chinese medicine (TCM) are widely used to improve the curative effect of exercise-induced knee injuries [5–8]. TCM is uniquely advantageous in the treatment of knee injuries or knee osteoarthritis with less pain, higher efficacy, and fewer adverse effects. In the present study, Chinese medical treatments such as Tuina, acupuncture, and Chinese herbal compresses were used to delay the degeneration of articular cartilage and promote repair by improving local microcirculation, regulating abnormal cytokine levels, and inhibiting matrix-degrading enzymes. Previously, combined treatment of rehabilitation therapy and nonsteroidal antiinflammatory drugs was usually adopted to relieve patients' symptoms. Nonsteroidal antiinflammatory drugs reduce the metabolism of arachidonic acid into inflammatory mediators such as prostaglandins, prostacyclins, and thromboxanes by inhibiting epoxygenase in the body, thereby alleviating joint swelling and pain by mitigating the inflammatory phenomena such as congestion and exudation in the synovial membrane at the knee joint injury. It is a nonspecific symptomatic drug for arthritis and inhibits prostaglandin synthesis in the hypothalamic thermoregulatory center, with antiinflammatory, peripheral analgesic, and antipyretic effects. However, long-term use of nonsteroidal antiinflammatory drugs is associated with an increased risk of cartilage damage. Glucosamine hydrochloride, mostly used for elderly knee osteoarthritis, promotes the articular cartilage mechanism and the biosynthesis of articular cartilage proteins, thereby inhibiting the matrix metalloproteinase cell growth factor that damages the cartilage [9–12]. Osteoarthritis of the knee is a degenerative disease in which primary or secondary degenerative changes in the articular cartilage of the knee joint occur due to various causes (trauma, persistent strain) and are accompanied by subchondral bone growth, resulting in gradual destruction and deformity of the joint surface and compromised knee joint function. The affected area of knee osteoarthritis is similar to that of a sports knee injury. Exercise-induced knee injuries are also prone to cartilage damage, and chondrocytes are difficult to regenerate once the articular cartilage is damaged. Glucosamine hydrochloride can inhibit the loss of glycoproteins within the cartilage matrix in knee osteoarthritis, avoid cartilage softening in the surface layer of the joint, and suppress the action of matrix metalloproteinase cell growth factor. Studies on the effects of glucosamine hydrochloride on exercise-induced knee injuries are scarcely reported, and this study was therefore conducted to provide new clinical insights into the treatment. Accordingly, the clinical data of 96 patients with exercise-induced knee injuries who were admitted to our hospital from February 2019 to February 202 were retrospectively analyzed to evaluate the application value of comprehensive rehabilitation therapy combined with glucosamine hydrochloride for exercise-induced knee joint injury and its effect on knee joint function.

RETRACTED

## 2. Research Process

### 2.1. Research Object

#### 2.1.1. Diagnostic Criteria

① The knee joint injury was caused during exercise, and a clear history of trauma; ② after injury, there were symptoms such as joint swelling, pain, locked knee, restricted movement, and noise during movement; ③ patients with joint space tenderness, McMurray test (+), patellar tap (+), and knee swing test (+); and ④ *magnetic resonance imaging* examination of the meniscus showed no tears or other injuries.

#### 2.1.2. Inclusion Criteria

With reference to the Guidelines for the Treatment of Osteoarthritis (2018 Edition) [13], patients were enrolled within 12 hours after the injury, without a history of serious knee trauma or fracture, with clear and complete clinical medical records, without use of glucocorticoids or nonsteroidal antiinflammatory drugs in the past three months, and who provided written informed consent were included.

#### 2.1.3. Exclusion Criteria

Patients with rheumatoid arthritis, gouty arthritis, ankylosing spondylitis, and psoriatic arthritis, with local skin ulceration of the knee joint, with lower limb fractures, knee cruciate ligament, and collateral ligament rupture, symptoms that seriously compromise the patient's limb motor function, during pregnancy or lactation, and with internal deformity of the knee exceeding 10°, external deformity exceeding 15°, and active knee flexion and extension mobility less than 80° were excluded.

### 2.2. Grouping

All patients were assigned at a ratio of 1 : 1 with matched general information to a control group (*n* = 45) receiving comprehensive rehabilitation therapy and an experimental group (*n* *=* 51) given comprehensive rehabilitation therapy combined with glucosamine hydrochloride tablets. This study was a retrospective study that only collected clinical data of patients without interfering with the treatment protocols of patients and was approved and supervised by the ethics committee of the second hospital in Tangshan, Approval No. 97991/7. This study was reported in compliance with the Strengthening the Reporting of Observational Studies in Epidemiology (STROBE) statement, and the collected data were archived in the case room, without independent recollection of patients. The sample size was determined according to the hospital sample survey case-control study method, with an estimated prevalence of 5%, a relative error of 15% for sampling, and a design efficiency deff set at 2.0 with reference to the Osteoarthritis Treatment Guidelines (2018 edition) and other similar large health surveys, with a 95% confidence interval, Za = 1.96, and a 10% data incompleteness rate. After calculation, a sample size of 40–50 was determined.

RETRACTED

### 2.3. Intervention Methods

Control group: comprehensive rehabilitation therapy mainly includes massage, acupuncture, and TCM herbal application. (1) Massage: the acupoints of the Zuyangming Meridian and Zuyangming Meridian of the patients were massaged to relax muscles and collaterals. The painful area of the patient was massaged to dredge the Qi of the muscles. The tendon correction technique was used to loosen the knots around the knee joint to correct the position of the tendons. Massage techniques such as pinching and tapping were adopted to relax the fascia and muscles around the calf and thigh. The malaxation method was used to relax the related muscle groups around the knee joint [13–15]. (2) Acupuncture: with the patient in a supine or sitting position, after the sterilization of the acupuncture site with 75% alcohol, disposable sterile acupuncture needles (specification: 0.30 mm × 40 mm) were used to pierce the acupoints of Xiyan, Weiyang, Weizhong, Ashi, Liangqiu, Yinlingquan, Yanglingquan, Heding, and Heyang on the affected limb. The needles were swiftly inserted at 25–30 mm depth through the method of neutral supplementation and draining and then connected with an electroacupuncture instrument (model: G6805-2A), with a dilatational wave persisting for 30 minutes and an appropriate current intensity that causes local muscle tremor. Acupuncture was performed once a day. (3) TCM herbal application: patients received one tape of Yunnan Baiyao Antiinflammatory Analgesic Ointment Tape (Yunnan Baiyao Group Co., Ltd., National Medical Products Administration Approval number Z53020756) on the injured knee joint daily. The duration of treatment was 8 weeks.

Experimental group: on the basis of the control group, the patients received 0.75 g of glucosamine hydrochloride tablets (Aomei Pharmaceutical Co., Ltd., National Medical Products Administration Approval number HC20140007) through oral administration, twice daily after breakfast and dinner. The duration of the treatment was 8 weeks.

### 2.4. Observational Indicators

General information: the age, gender, course of the disease, body mass index (BMI), affected side, and exercise events of the two groups of patients were collected and statistically processed to calculate the differences between the groups.

Clinical efficacy: clinical efficacy was determined based on the “Diagnosis and Efficacy Criteria for TCM Diseases” [16]. Cured: the knee joint moves normally with completely restored joint function. Significantly effective: joint swelling and pain disappeared, tenderness was relieved, and knee joint function was basically restored. Effective: the joints were swollen and painful, and partial joint function was basically restored. Ineffective: no significant improvement in the conditions was observed. Objective effective rate = (cured + significantly effective + effective)/total × 100%.

RETRACTED

Pain score: the visual analogue scale (VAS) was used to evaluate the degree of pain before and after the treatment. A score of 0 means no pain, and a score of 10 represents unbearable pain, with 0–2 for comfortable, 3–4 for mildly uncomfortable, 5–6 for moderately uncomfortable, 7–8 for severely uncomfortable, and –910 for extremely uncomfortable. The VAS scores of the two groups of patients were analyzed.

C-reactive protein: 4 ml of synovial fluid was drawn for the determination of C-reactive protein level by using the enzyme-linked immunosorbent method with an American whole-series East Microplate Reader (Model: Bio-Bad).

Walking ability: 0 points, patients had no restrictions on walking; 1 point, patients with restricted walking ability but could walk over 1 km. 2 points, patients could walk about 1 km or 15 minutes. 3 points, patients could walk 500–900 m or 8–15 min. 4 points, patients could only walk 300–500 m. 5 points, patients could only walk 100–300 m. 6 points, patients failed to walk more than 100 m. The score was added with 1 point if the patients walked with one crutch and 2 points with two crutches.

Lysholm knee score: the scale includes 8 evaluation dimensions of claudication, support, pain, swelling, locked knee, climbing, squatting, and instability. The maximum score is 100 points. The higher the score, the better the knee joint function of the patient.

Five-times-sit-to-stand-test (FTSST) : the participant sat on a 43 cm high chair without armrests, with feet on the ground, not leaning on the back of the chair, with arms crossed in front of the chest. After hearing the instruction, the participant completed the 5 rising and sitting movements as fast as possible. The time (in seconds) taken to complete the five movements was recorded. During the test, the participant was required to cross their hands in front of their chest and to stand with their knees fully extended. The FTSST provides good retest reliability [11].

### 2.5. Statistical Processing

The data obtained in this study were processed by the software SPSS 21.0, and the graphics plotting was processed using the GraphPad Prism 7 (GraphPad Software, San Diego, USA) software. The research data included count data and measurement data. Count data were expressed as [n (%)] and processed by the X^2^ test, and Fisher's exact test was performed when the theoretical frequency was <5. The measurement data were expressed as $\bar{x}$ ± *s*. Two independent sample *t*-test was used for intergroup comparisons, and a paired *t*-test was used for intragroup comparisons. *P* < 0.05  was used as a cut-off for statistical significance.

RETRACTED

## 3. Results

### 3.1. Patient Characteristics

The patient characteristics of the two groups, such as age, course of disease, BMI, gender, affected side, and exercise, were comparable (*P* > 0.05) (Table 1).

### 3.2. Clinical Efficacy

In the control group, there were 6 (13.33%) cases of ineffective, 11 (24.44%) cases of effective, 15 (33.33%) cases of significantly effective, and 13 (28.89%) cases of cured, with an overall efficacy of 86.67%. In the experimental group, there was 1 (1.96%) case of ineffective, 10 (19.61%) cases of effective, 15 (29.41%) cases of significantly effective, and 25 (49.02%) cases of cured, with an overall efficacy of 98.04%. The experimental group showed a significantly higher clinical efficacy as compared to the control group (*P*=0.048) (Figure 1).

### 3.3. VAS Score

Before treatment, the VAS scores of the control group and the experimental group were 4.48 ± 1.30 and 4.52 ± 1.29 points, respectively. After treatment, the VAS scores of the control group and the experimental group were 1.43 ± 0.32 and 1.15 ± 0.25 points, respectively. After the treatment, the VAS scores of the two groups showed a decline, with a lower result in the experimental group (*P* < 0.001), as shown in Table 2.

### 3.4. C-Reactive Protein Levels

Before treatment, the C-reactive protein levels of the control group and the experimental group were 1.80 ± 0.31 and 1.83 ± 0.29 mg/L, respectively. After treatment, the VAS scores of the control group and the experimental group were 1.65 ± 0.26 and 1.50 ± 0.19 mg/L, respectively. After the treatment, the C-reactive protein levels of both groups decreased, with lower levels being observed in the experimental group compared with the control group (*P* < 0.05). See Table 3.

### 3.5. Walking Ability

The walking ability scores of the control group before and after treatment were 5.43 ± 1.14 points and 1.86 ± 0.37 points. The walking ability scores of the experimental group before and after treatment were 5.52 ± 1.16 points and 1.25 ± 0.23 points. Patients in the experimental group had a lower walking ability score than those in the control group after the treatment (*P* < 0.001), as shown in Figure 2.

### 3.6. Lysholm Score

The Lysholm scores of the control group before and after the treatment were 49.84 ± 11.12 points and 77.86 ± 12.53 points. The Lysholm scores of the experimental group before and after the treatment were 50.43 ± 11.64 points and 86.48 ± 16.73 points. Results in Figure 3 demonstrated remarkably higher post-treatment Lysholm scores in the experimental group than in the control group (*P* < 0.001).

RETRACTED

### 3.7. FTSST

Before treatment, the FTSST of the control group and the experimental group were 22.38 ± 4.05 and 22.29 ± 3.96 s, respectively. After treatment, the VAS scores of the control group and the experimental group were 17.11 ± 3.30 and 13.98 ± 2.87 s, respectively. Strong evidence of shorter FTSST for the experimental group than the control group (*P* < 0.05) was found in Table 4.

## 4. Discussion

Exercise-induced knee injury mainly refers to the injuries of knee joint tissue structures or functions that may occur in any sports event, with manifestations of pain, swelling, restricted knee movement, and symptoms such as redness, swelling, and hot pain in the acute stage. A cold compress can stop the bleeding, reduce swelling, and relieve pain by promoting vasoconstriction, reducing local congestion, and lowering tissue temperature [17–20]. Clinical treatment of exercise-induced knee injuries is classified into nondrug treatment and drug treatment. Nondrug therapy mainly employs comprehensive rehabilitation therapies such as massage, acupuncture, and Chinese medicine herbal application to mitigate knee joint pain and promote the recovery of knee joint function. Nonsteroidal antiinflammatory drugs, analgesics, intraarticular injections (such as sodium hyaluronate and glucocorticoids), and chronically acting drugs that relieve symptoms (such as glucosamine hydrochloride) are mostly used in drug therapy [20–23]. Glucosamine hydrochloride is an amino monosaccharide obtained from chitin by hydrochloric acid hydrolysis. It directly replenishes the cartilage matrix, prevents cartilage degradation, stimulates chondrocyte production of proteoglycans, and inhibits the production of collagenase, superoxide radicals, and phospholipase A2, thereby protecting articular cartilage tissue and facilitating cartilage regeneration. However, there are few reports investigating the effect of glucosamine hydrochloride on exercise-induced knee joint injuries.

Results of the present study found that the efficacy of the experimental group was significantly higher than that of the control group (*P* < 0.05), indicating a promising therapeutic effect of the combination of glucosamine hydrochloride with comprehensive rehabilitation therapy, which may be attributed to the fact that the biosynthesis of mucopolysaccharides increases the intake of skeletal calcium, improves the metabolic function of cartilage tissue, and enhances the viscosity of the synovial fluid through the stimulation of glucosamine hydrochloride. This result was consistent with the results of Bruyère [24] et al. After the treatment, the VAS scores and c-reactive protein of the two groups showed a decline, with a lower result in the experimental group than in the control group (*P* < 0.05), suggesting that the combination therapy prominently abates the pain of exercise-induced knee joint injuries. Acupoint massage and acupuncture regulate joint function, promote blood circulation, and mitigate muscle tension. Moreover, glucosamine hydrochloride relieves pain and significantly reduces the level of inflammatory factors in the joint cavity. The Lysholm knee scores were increased in the two groups after the treatment, with a higher score obtained in the experimental group in contrast to the control group (*P* < 0.05). After the treatment, patients of both groups had a shorter FTSST, with better outcomes obtained in the experimental group than in the control group (*P* < 0.05). The results further confirmed that glucosamine hydrochloride improves the repair capacity of chondrocytes and promotes cartilage matrix restoration, thereby relieving joint pain and improving joint movement.

RETRACTED

## 5. Conclusion

Comprehensive rehabilitation therapy plus glucosamine hydrochloride effectively improves the clinical efficacy of exercise-induced knee joint injuries and enhances knee joint function rehabilitation. The limitations of this study are as follows: (1) the study is a retrospective analysis study, and the relatively short follow-up duration results in insufficient long-term treatment data; and (2) glucosamine hydrochloride has good drug resistance, but it is associated with slight gastrointestinal discomfort. In clinical application, it can be used in combination with nonsteroidal antiinflammatory drugs according to the patient's condition. To address the limitations of this study, a multicenter randomized prospective analysis with a large sample will be conducted in the future to extend the study follow-up time and obtain long-term clinical efficacy data. The molecular mechanisms of the drug targets were also investigated to obtain biomarker targets for adverse drug reactions.

## Figures and Tables

**Figure 1:** Comparison of the clinical efficacy of the two groups of patients (%). Note: The abscissa represents the clinical efficacy observation index, and the ordinate represents the percentage.

**Figure 2:** Comparison of the walking ability scores of the two groups of patients ($\bar{x}$ ± *s*). Note: The abscissa indicates before and after treatment, and the ordinate indicates the score. The walking ability scores of the control group before and after treatment were: (5.43 ± 1.14) points and (1.86 ± 0.37) points. The walking ability scores of the experimental group before and after treatment were: (5.52 ± 1.16) points and (1.25 ± 0.23) points. There is a significant difference in the walking ability scores between the two groups of patients after treatment (*t* = 9.821, ^*∗∗∗*^*P* < 0.001).

RETRACTED

**Figure 3:** Comparison of Lysholm scores between the two groups of patients ($\bar{x}$ ± *s*). Note: The abscissa indicates before and after treatment, and the ordinate indicates the score. The Lysholm scores of the control group before and after the treatment were: (49.84 ± 11.12) points and (77.86 ± 12.53) points. The Lysholm scores of the experimental group before and after the treatment were: (50.43 ± 11.64) points and (86.48 ± 16.73) points. A significant difference in Lysholm scores between the two groups of patients after the treatment (*t* = 2.836, ^*∗*^*P*=0.006).

**Table 1:** Comparison of general information of the two groups of patients.

Indexes	Control group (*n* = 45）	Experimental group (*n* = 51)	*X* ^2^/*t*	*P*
Age (year)	32.42 ± 8.15	33.07 ± 8.29	0.386	0.700
Course of disease (h)	6.42 ± 1.44	6.51 ± 1.52	0.297	0.767
BMI (kg/m^2^)	22.84 ± 1.96	22.83 ± 1.91	0.025	0.980
Gender			0.041	0.840
Male	15 (33.33)	18 (35.29)		
Female	30 (66.67)	33 (64.71)		
Affected side			0.400	0.527
Left knee	14 (31.11)	19 (37.25)		
Right knee	31 (68.89)	32 (62.74)		
Exercise			0.216	0.642
Basketball	11 (24.44)	11 (21.57)		
Martial arts competition	8 (17.78)	11 (21.57)		
Ice and snow sports	13 (28.89)	15 (29.41)		
Weightlifting	6 (13.33)	7 (13.73)		
Badminton	2 (4.44)	3 (5.88)		
Long jump	5 (11.11)	4 (7.84)		

**Table 2:** Comparison of the VAS scores of the two groups of patients ($\bar{x}$ ± *s*).

Groups	Before treatment	After treatment	*t*	*P*
Control group (*n* = 45)	4.48 ± 1.30	1.43 ± 0.32	15.282	<0.001
Experimental group (*n* = 51)	4.52 ± 1.29	1.15 ± 0.25	18.316	<0.001
*T*	3.564	4.805		
*P*	0.545	<0.001		

**Table 3:** Comparison of C-reactive protein levels between the two groups of patients (mg/L, $\bar{x}$ ± *s*).

Detection time point	Control group (*n* = 45)	Experimental group (*n* = 51)	*t*	*P*
Before treatment	1.80 ± 0.31	1.83 ± 0.29	4.567	0.364
After treatment	1.65 ± 0.26	1.50 ± 0.19	3.253	0.002
*T*	2.487	6.797		
*P*	0.015	<0.001		

**Table 4:** Comparison of FTSST between the two groups of patients (*s*, $\bar{x}$ ± *s*).

Detection time point	Control group (*n* = 45)	Experimental group (*n* = 51)	*t*	*P*
Before treatment	22.38 ± 4.05	22.29 ± 3.96	7.564	0.167
After treatment	17.11 ± 3.30	13.98 ± 2.87	4.971	<0.001
*T*	6.767	12.134		
*P*	<0.001	<0.001		

## Data Availability

No data were used to support this study.
